# Malignancy risk of gastrointestinal stromal tumors evaluated with noninvasive radiomics: A multi-center study

**DOI:** 10.3389/fonc.2022.966743

**Published:** 2022-08-16

**Authors:** Yun Wang, Yurui Wang, Jialiang Ren, Linyi Jia, Luyao Ma, Xiaoping Yin, Fei Yang, Bu-Lang Gao

**Affiliations:** ^1^ Affiliated Hospital of Hebei University/Hebei University (Clinical Medical College), Baoding, China; ^2^ Tangshan Gongren Hospital, Tangshan, China; ^3^ General Electric Pharmaceutical Co., Ltd, Shanghai, China; ^4^ Xingtai People’s Hospital, Xingtai, China; ^5^ Medical Imaging Department, The First Affiliated Hospital of Hebei North University, Zhangjiakou, China

**Keywords:** gastrointestinal stromal tumors, traditional CT diagnosis, enhance different periods, radiomics, multiple centers

## Abstract

**Purpose:**

This study was to investigate the diagnostic efficacy of radiomics models based on the enhanced CT images in differentiating the malignant risk of gastrointestinal stromal tumors (GIST) in comparison with the clinical indicators model and traditional CT diagnostic criteria.

**Materials and methods:**

A total of 342 patients with GISTs confirmed histopathologically were enrolled from five medical centers. Data of patients wrom two centers comprised the training group (n=196), and data from the remaining three centers constituted the validation group (n=146). After CT image segmentation and feature extraction and selection, the arterial phase model and venous phase model were established. The maximum diameter of the tumor and internal necrosis were used to establish a clinical indicators model. The traditional CT diagnostic criteria were established for the classification of malignant potential of tumor. The performance of the four models was assessed using the receiver operating characteristics curve.

**Reuslts:**

In the training group, the area under the curves(AUCs) of the arterial phase model, venous phase model, clinical indicators model, and traditional CT diagnostic criteria were 0.930 [95% confidence interval (CI): 0.895-0.965), 0.933 (95%CI 0.898-0.967), 0.917 (95%CI 0.872-0.961) and 0.782 (95%CI 0.717-0.848), respectively. In the validation group, the AUCs of the models were 0.960 (95%CI 0.930-0.990), 0.961 (95% CI 0.930-0.992), 0.922 (95%CI 0.884-0.960) and 0.768 (95%CI 0.692-0.844), respectively. No significant difference was detected in the AUC between the arterial phase model, venous phase model, and clinical indicators model by the DeLong test, whereas a significant difference was observed between the traditional CT diagnostic criteria and the other three models.

**Conclusion:**

The radiomics model using the morphological features of GISTs play a significant role in tumor risk stratification and can provide a reference for clinical diagnosis and treatment plan.

## Introduction

Gastrointestinal stromal tumors (GISTs) are the most common mesenchymal tumors in the gastrointestinal tract of middle-aged and elderly (60-70 years old) patients. The common sites of GIST are stomach (50%-60%), small intestine (20%-30%), colorectal (5%-10%), and esophagus (< 5%) (1, 2). GISTs exhibit a specific malignant potential as well as early liver and abdominal metastasis. According to the National Institute of Health (NIH) 2008 standard (3), the risk of GIST can be divided into very low risk, low risk, medium risk, and high risk. Typically, GISTs with a very low or low risk are classified as potential malignant, whereas those with a medium or high risk are classified as malignant. Because of the heterogeneity, different individuals considered different malignant potentials with varied treatment approaches in the same GIST lesion. Clinically, the potentially malignant GISTs are treated as a benign tumor, whereas malignant GISTs are treated with imatinib mesylate and other drugs before or after the operation to prevent recurrence or metastasis (4). The gold standard for malignant diagnosis of GIST is based on the pathological results, including tumor size, mitotic count and tumor site (**Table 1**) (3, 5). In order to obtain pathological samples of tumor for risk grading and evaluation of the tumor, a puncture biopsy is essential. However, this is an invasive method and might lead to tumor cell metastasis and tumor bleeding. Therefore, risk classification of the tumor should be obtained at the earliest time possible for selection of an appropriate clinical treatment plan. Although computed tomography (CT) is of a great value in detecting GISTs (6), it is still difficult to judge the malignant potential of tumors due to lack of understanding of the images or unclear tumor signs.

**Table 1:** NIH 2008 criteria for risk stratification of GIST recurrence after surgery.

Risk category	Tumor size (cm)	Mitotic index (per 50 HPF)	Location
Very low risk	≤ 2.0	≤ 5.0	Any
Low risk	2.1-5.0	≤ 5.0	Any
Intermediate risk	≤ 5.0	6-10	Gastric
	5.1-10.0	≤ 5.0	Gastric
High risk	>10.0	Any	Any
	Any	>10	Any
	>5.0	>5	Any
	≤ 5.0	>5	Non-gastric
	5.1-10.0	≤ 5	Non-gastric

GIST, gastrointestinal stromal tumor; HPF, high-power field.

In recent years, rapid development in medical imaging analysis and imaging pattern recognition tools has promoted the development of a high-throughput quantitative feature extraction process, the radiomics, which converts images into exploitable data for analysis (7). This technique can be used to diagnose noninvasively the nature of lesions and ultimately assist the radiologist in making an accurate diagnosis. In the evaluation of the malignancy of GISTs, radiomics has been applied using data of ultrasound, magnetic resonance imaging, and CT (8–13). However, no studies have been performed wtih CT data in the arterial and venous phase to extract the radiomics features for evaluation of the malignancy of GISTs. The present study aimed to explore the radiomics diagnostic models of GIST with different degrees of risk based on the CT image data in the arterial phase and venous phase from five medical centers, with four models being estalibshed, including the arterial phase model, venous phase model, clinical indicators model, and traditional CT diagnostic criteria. The data in two centers were set up as the training group to reduce the sampling bias and to establish a more ubiquitous radiomics model than those in one center only, with the slice thickness of images as 5 mm (14). The diagnostic efficiency was also evaluated to find the best model to guide the correct clinical decision-making process.

## Materials and methods

### Patients

This retrospective study was approved by the Institutional Review Board of the Affiliated Hospital of Hebei University, and all patients had given their signed informed consent to participate. All methods were performed in accordance with the relevant guidelines and regulations. The data of CT images of 342 patients were collected from five medical centers from January 2015 to August 2021. Two centers were randomly selected and assigned to the training group, and the data of the other three centers were set up as the validation group.

The inclusion criteria were patients with GISTs confirmed by pathology, complete clinical and pathological data (lesion size, origin location, and risk classification), and standard dynamic enhanced CT scan at least 15 days before the operation. The exclusion criteria were patients with a previous history of other coexisting malignant tumors, neoadjuvant chemoradiotherapy before CT scan, and poor image quality precluding quantitative analyses. The selection process of patient cohorts is shown in **Figure 1**.

**Figure 1:** A flowchart shows selection of study population and exclusion criteria.

### CT scanning instruments and methods

The Discovery CT750 HD scanner (GE Medical Systems, Milwaukee, WI, USA), Toshiba Aquilion 64-slice spiral CT scanner (Tokyo harbor area, Japan), Philips 256-slice ICT scanner (Amsterdam, The Netherlands), and Philips brilliance 64-slice CT scanner (Amsterdam, The Netherlands) were used for CT scanning. After fasting for 6-8 h, the patient had warm water (500-1000 mL) 10 min before the examination with plain and enhanced abdominal scanning in the supine position. The scanning parameters were as follows: slice thickness 5 mm, pitch 0.9-1.0, scanning field 350 mm×350 mm, matrix 512×512, tube voltage 100–120 kV, tube current 160–300 mA, and X-ray tube rotation time 0.5–0.8 s. The contrast agent was injected through the elbow vein at a flow rate of 3.0–3.5 mL/s and a dose of 1.0–1.2 mL/kg body weight. The scanning time of the arterial phase, venous phase, and delayed phase was 30-35 s, 50-60 s, and 180 s, respectively, after injection of contrast agent. The CT images at the arterial and venous phase were selected for imaging analysis.

### Clinical data

The clinical data including age, gender of patients, and tumor location were collected based on pathological results. The imaging data including tumor maximal diameter and necrosis within the tumor lesion were collected based on CT imaging. In the malignant potential classification using the traditional CT diagnosis method, the CT images were assessed by five radiologists (with 19, 15, 10, 8 and 4 years of working experience, respectively) who were blinded to the pathological diagnoses in all cases. The tumor is divided into potentially malignant and malignant according to the CT image characteristics, including tumor size, location, shape, boundary, enhancement mode and degree, infiltration of peripheral organs, and lymph node enlargement (15–17). In disagreement, a consensus was reached after discussion.

### CT image segmentation

Two radiologists (physicians 1 and 2) with 10 years of experience in the abdominal imaging diagnosis applied the ITK-SNAP software (version 3.8.0, https://www.itksnap.org) to delineate the CT-enhanced images at the arterial and venous phases. The delineated areas included the tumor lesion as much as possible without inclusion of the surrounding normal tissues or other tissues in order to generate a two-dimensional (2D) region of interest (ROI) (**Figure 2**). The 2D ROI was then recombined to generate a 3D volume of interest (VOI) for subsequent image feature extraction and analysis.

**Figure 2:** Imaging segmentation of gastrointestinal stromal tumors (GIST) on computed tomography (CT) imaging. **(A)** Two-dimensional (2D) CT arterial phase image of potential malignant GIST. The tumor is quasicircular and uniformly enhanced. The red outline is the boundary drawn by radiologists to show the tumor. **(B)** 2D segmentation of the tumor. **(C)** 3D segmentation of the tumor lesion. **(D)** 2D CT arterial phase image of malignant GIST with irregular shape and uneven internal enhancement of the tumor. The red outline is the boundary drawn by radiologists to show the tumor lesion. **(E)** 2D segmentation of the tumor. **(F)** 3D segmentation of the tumor.

### Radiomic feature extraction and selection

CT images with different scanning parameters were preprocessed. The linear interpolation method was used to resample the image to 1×1×1 mm^3^, attempting to alleviate the influence of different layer thicknesses. The image gray was discretized, the bin width was set to 25, and the image filtering process was used to highlight different bandwidth signals and prevent the noise in ROI from interfering with texture information. Parameters σ 3 and 5 of Laplace of Gaussian (LOG) filter and wavelet were used. After wavelet decomposition, eight categories of information of the filtered features were obtained from the original set of feature information. The preprocessed image and the outlined ROI files were imported into the platform of “pyradiomics” for radiomics feature extraction, and two sets of image filtering were utilized. A total of 1037 features were generated from the histogram (18 features), morphological feature (14 features), texture feature of gray level co-occurrence matrix (GLCM, 24 features), gray-level run-length matrix (GLRLM, 16 features), gray-level size zone matrix (GLSZM, 16 features), gray-level dependence matrix (GLDM, 14 features), and neighborhood gray-tone difference matrix (NGTDM, 5 features).

In order to prevent overfitting risk, it was necessary to reduce the dimension of data features and select those with the best efficiency and most research significance. A total of 20 important features were selected using the minimum redundancy maximum relevance feature selection (mRMR) based on relevant references in the literature to prevent distortion of model (18–20). Subsequently, the least absolute contraction selection operator (LASSO) was used to further eliminate collinear features, and 5 features in the arterial phase and 11 features in the venous phase were kept.

### Radiomics models building

The arterial phase model and venous phase model of radiomics: After feature selection, 5 features of arterial phase and 11 features of venous phase were used to retain the minimum Akaike information criterion (AIC) feature set by the multifactor stepwise regression.

Clinical indicators model of radiomics: The clinical indicators of the tumor diameter (>5 cm) and internal necrosis were used as clinical features. The model was established by multiple regression analysis with the maximal diameter of the tumor and presence of necrosis as the feature of the model and benign or malignant nature as the goal.

Traditional CT diagnostic criteria of radiommics: According to the consolidated GIST CT diagnosis results of the five evaluating radiologists, the traditional CT diagnostic criteria were used for classification of the malignant potential of the tumors.

### Sample size estimation

In the training group, 196 consecutive patients were enrolled in two centers between January 2016 and December 2019. The training cohort contained 58 low-risk GIST patients and 138 high-risk patients. There were in total 2 predictors in our model (internal tumor necrosis and tumor diameter), making an event-per-predictor ratio of large than 10, which fell in the range of 5-9 in the rule of thumb for event-per-predictor in logistic regression models (21). In the validation group, the validation sample size was determined according to the method of sample size estimation for clinical research by Chow and colleagues (22), with the sample size being calculated to test whether the means of two groups were significantly different. Based on this method, the mimimal number of validation sameples were 14 (low-risk) and 36 (high-risk) in the group with the desired two-sided significance level of α=0.05 and power of 1-β=95%.

### Statistical analysis

All statistical analyses were performed using the R software (version 4.1.0, www.rporject.org). Measurement data were presented as median [Q1-Q3] if in non-normal distribution and tested with the Mann-Whitney U test, and enumeration data were expressed as numbers of cases (n) or percentage (%) and tested with the Chi square test. The non-normal distribution data of measurement were presented as median and interquartile range and tested with the Chi square test. Interclass and intraclass correlation coefficients (ICC) were used to evaluate the consistency of imaging features within and between observers. A total of 30 cases of CT images were randomly selected for ROI segmentation by physicians 1 and 2. One week later, physician 1 repeated the same steps, with an ICC >0.75 indicating good consistency in feature extraction. The segmentation of the remaining image was also completed by physician 1. The receiver operator characteristic (ROC) curve was used to evaluate the predictive efficacy of the malignant potential of GISTs in the models. The larger the area under the ROC curve (AUC), the higher the diagnostic efficiency. The AUC, accuracy, sensitivity, and specificity were calculated, and the ROC curves were assessed by the Delong test. All indexes were evaluated separately in the training and validation groups. Two-side *P*<0.05 was set as statistic significant.

## Results

### Clinical characteristics

According to the inclusion and exclusion criteria, data from 342subjects with GISTs, including 156 (45.6%) males and 186 (54.4%) females with an age range 33-82 (62.00 [54.00-69.00]) years, were collected. The GIST lesion was in the stomach in 226 (66.1%) cases and of a non-stomach location in 106 (33.9%), including 104 (30.4%) cases with potential malignancy (26 cases with an extremely low risk and 78 cases with a low risk) and 238 (69.6%) cases with malignancy (86 cases with a moderate risk and 152 cases with a high risk). According to the traditional CT diagnosis criteria for GISTs, 130 (38.0%) cases exhibited potential malignancy, whereas 212 (62.0%) cases were malignant. The diameter of the tumors was 1-24 (mean 6.9 ± 4.1) cm, with the tumor maximal diameter ≥5 cm in 214 (62.6%) cases and <5 cm in 128 (37.4%). Internal necrosis was presented in 176 (51.5%) cases. In the radiomics model, the patients were divided into the training (n=196) and validation (n=146) group (**Table 2**), with no significant (P>0.05) difference in the age, gender, malignancy potential, CT diagnostic grade, tumor maximal diameter >5 cm, and internal necrosis between the training and validation groups.

**Table 2:** Clinical data of the training and validation groups.

Variables	Training (n=196)	Validation (n=146)	P
Gender			0.181^1^
Female	112	74	
Male	84	72	
Age [median, Q1-Q3]	62.000 [56.000-69.000]	63.000 [52.000-69.000]	0.508^2^
Real malignant potential			0.793^1^
Potential malignancy	58(29.6%)	46(31.5%)	
Malignant	138(70.4%)	100(68.5%)	
Traditional CT classification			0.990^1^
Potential malignancy	64	48	
Malignant	132	98	
Maximal diameter ≥5 cm			0.847^1^
No	72	56	
Yes	124	90	
Internal necrosis			0.006^1^
No	82	84	
Yes	114	62	

Q1,First quarter; Q3, Three quarter; ^1^ Chi square test; ^2^Mann-Whitney U test.

### Univariable and multivariable analysis

In univariate analysis of GIST parameters, the tumor maximal diameter and internal necrosis were statistically significant (P<0.001) between potentially malignant and malignant GISTs (**Table 3**). Using the significant variables from the univariate analysis as inputs, multivariate logistic regression analysis showed that lesion diameter ≥ 5cm (coeficient 3.264, OR 26.17 (7.832-109.083), P<0.001) and lesion internal necrosis (coefficient 2.014, OR 7.491 (1.969-31.461), P=0.003) were independent factors for predicting malignant GIST.

**Table 3:** Univariable analysis of potentially malignant and malignant GISTs.

Variables	Training group			Validation group		
	Potentially malignant (n=104)	Malignant (n=238)	*P*	Potentially malignant (n=104)	Malignant (n=238)	*P*
Sex			0.910^1^			0.316^1^
Female	34(58.621%)	78(56.522%)		20(43.478%)	54(54.000%)	
Male	24(41.379%)	60(43.478%)		26(56.522%)	46(46.000%)	
Age[meadian, Q1-Q3]	61.000 [58.000-68.000]	63.000 [55.000-69.000]	0.683^2^	64.000 [54.250-71.500]	62.500 [51.000-68.000]	0.172^2^
Diameter ≥5 cm			<0.001^1^			<0.001^1^
No	54(93.103%)	18(13.043%)		42(91.304%)	14(14.000%)	
Yes	4(6.897%)	120(86.957%)		4(8.696%)	86(86.000%)	
Internal necrosis			<0.001^1^			<0.001^1^
No	54(93.103%)	28(20.290%)		46(100.000%)	38(38.000%)	
Yes	4(6.897%)	110(79.710%)		0(0.000%)	62(62.000%)	

GIST, gastrointestinal stromal tumors; Q1, First quarter; Q3, Three quarter; ^1^ Chi square test; ^2^ Mann-Whitney U test.

### ICC of radiomic features

A total of 1037 radiomics features with good consistency (mena ICC 0.95, range 0.75-1.0) were selected, whereas 95 features with bad consistency (ICC <0.75) were removed.

### Predictive performance of radiomics models

After feature selection, the radiomics features of the arterial and venous phases only preserved the morphological features. ROC curve analyses were performed for the arterial and venous phase models, clinical indicators model, and traditional CT diagnostic criteria (**Figure 3**), with a good calibration demonstrated in the arterial and venous phase models (**Figure 4**). The Radscore distribution of the arterial and venous phase models in the training and validation group were shown in **Figure 5**.

**Figure 3:** Receiver operating characteristics (ROC) curve analysis for different models in the training group **(A)** and validation group **(B)**.

**Figure 4:** Calibration curve for the arterial phase model, venous phase model, clinical indicators model and the traditional CT diagnostic criteria. The calibration of the four models was depicted by the calibration curve in terms of the agrement between the predicted risks of gastrointestinal stromal tumors (GISTs) and the actual results based on the modified criteria. The grey line represents an ideal prediction, and the other lines represent the predictive performance of the models. The closer the fit of the purpole line to the ideal line, the better the prediction.

**Figure 5:** The distribution of arterial and venous phase model radscore between patients suffered from malignant and potiential malignant tumors in the training group **(A, B)** and the validation group **(C, D)**.

In the ROC curve analyses for the training group, the AUC, accuracy, sensitivity, and specificity for grading tumor malignancy were 0.930 (95%CI: 0.895-0.965), 0.888, 0.928, and 0.793, respectively, for the arterial phase model; 0.933 (95%CI: 0.898-0.967), 0.857, 0.855, and 0.862, respectively, for the venous phase model; 0.917 (95%CI: 0.872-0.961), 0.918, 0.913, and 0.931, respectively, for the clinical indicators model;, and 0.782 (95%CI: 0.717-0.848), 0.806, 0.841, and 0.724, respectively, for the traditional CT diagnostic criteria. In the validation group, the AUC, accuracy, sensitivity, and specificity were 0.960(95%CI: 0.930-0.990), 0.932, 0.920, and 0.957, respectively, for the arterial phase model; 0.961 (95%CI: 0.930-0.992), 0.932, 0.920, and 0.957, respectively, for the venous phase model; 0.922 (95%CI: 0.884-0.960), 0.890, 0.880, and 0.913, respectively, for the clinical indicators model; and 0.768 (95%CI: 0.692-0.844), 0.795, 0.840 and 0.696, respectively, for the traditional CT diagnostic criteria (**Table 4**).

**Table 4:** Effectiveness of radiomics models in the grading of GIST malignancy.

Model	Training group(n=196)				Validation group(n=146)			
	AUC	Accuracy	Sensitivity	Specificity	AUC	Accuracy	Sensitivity	Specificity
A	0.930	0.888	0.928	0.793	0.960	0.932	0.920	0.957
V	0.933	0.857	0.855	0.862	0.961	0.932	0.920	0.957
Clinical	0.917	0.918	0.913	0.931	0.922	0.890	0.880	0.913
CT	0.782	0.806	0.841	0.724	0.768	0.795	0.840	0.696

GIST, gastrointestinal stromal tumor; AUC, area under the receiver operator characteristic curve; A, arterial phase model; V, venous phase model; Clinical, clinical indicators model; CT, traditional CT diagnostic criteria.

Comparison of the AUC values in grading tumor malignancy between different models using the Delong test was performed (**Table 5**). No significant (P>0.05) difference was detected in the AUC between the arterial and venous phase models, and clinical indicators model, whereas significant (P<0.01) differences were detected between the traditional CT diagnostic criteria (CT) and any of the other three models. The AUC value was significantly (P<0.01) better in the arterial phase model, venous phase model, and clinical indicators model than that in the traditional CT diagnostic criteria.

**Table 5:** Comparison of AUC results among models by the Delong test.

Model	Training group	Validation group
	*P*	*P*
A-V	0.879	0.897
A-Clinical	0.590	0.013
V-Clinical	0.439	0.013
A-CT	<0.001	<0.001
V-CT	<0.001	<0.001
Clinical-CT	<0.001	<0.001

AUC, area under the receiver operator characteristic curve; A, arterial phase model; V, venous phase model; Clinical, clinical indicators model; CT, traditional CT diagnostic criteria.

## Discussion

This study investigated the value of radiomics models in grading tumor malignancy of GISTs using enhanced CT imaging data from five medical centers, and four radiomics models were established based on the morphological features of the arterial and venous phase, clinical indicators, and traditional CT diagnostic criteria for GISTs. The models of the arterial phase, venous phase, and clinical indicators were significantly better than the traditional CT diagnostic criteria in grading the tumor malignancy of GISTs.

After studying CT venous phase images and radiomics features of GISTs in 222 cases including one training group (n=130) and one validation group (n=92) in the raiomics, Chen et al. (9) found that the radiomics features combined with clinical indicators and traditional CT characteristics were more effective in judging the malignant potential of GISTs as compared to the clinical indicators or traditional CT characteristic models. Through investigating 339 cases of GISTs from four centers including the training group (n=148), internal verification group (n=41), and external validation group (n=150), Zhang et al. (23) found that the radiomics features of enhanced CT were significantly correlated with the expression of Ki-67 in GISTs and that the tumor size had the highest prediction accuracy of Ki-67 expression. Wang et al. (24) established a radiomics model to predict the malignant potential and mitotic count of GISTs by analyzing the portal venous-phase images of 333 GIST cases, and it was also found that the combination of radiomics features, subjective CT examination results, and clinical indicators could be used to realize individualized risk prediction and improve the diagnostic level. However, these studies only selected the venous phase of GIST images with enhanced scanning as the research object, and no studies have investigated the difference in the radiomics characteristics of GISTs between the arterial phase and venous phase. Moreover, the data of the training group were from one single center, lacking multicenter data and consequently efficiency for generalization.

The texture performance of enhanced CT images at different periods varies, and to set up an appropriate radiomics model, it is crucial to select the texture features at different enhancement phases such as those of the arterial phase and venous phase. Several investigators have studied the CT enhancement degree of GIST, albeit different in the conclusions (1, 25–30). With the increase of GIST risk stratification, some researchers had found a declining trend in the CT value at each phase of enhanced scanning (28), whereas others had revealed that the degree of GIST enhancement was not related to risk classification (16). In addition, some investigators (17) had demonstrated that the GIST of the small intestine was highly malignant, with the tumor enhancement degree equal to that of adjacent intestinal wall. In case of an unclear correlation between tumor risk and CT enhancement degree, the radiomics features of CT images at different enhancement periods were used to stratify the GIST risk. Liu et al. (1) evaluated 78 patients with GISTs and found significant differences in the CT texture parameters with different GIST risks between the arterial phase and venous phase. Feng et al. (25) found that the entropy value at the venous phase was more accurate in distinguishing low-risk small bowel GIST from medium- and high-risk small bowel GIST as compared to that at the arterial phase. Also, some studies established radiomics models based on the CT arterial phase images (30) or venous phase images (29) so as to provide a noninvasive detection method for prediction of potential malignancy and malignancy of the GIST. Our study was based on GIST data from multicenters, and after extracting and selecting the radiomic features of the arterial and venous phases, only one morphological feature remained: the maximal diameter of the tumor. With only one morpholigcal feature left, good consistency could be easily obtained in the tumor delineation process, with similar efficiency in the arterial phase and venous phase features. The fact that there were no other radiomics features left could be attributed to the GIST data from multiple centers. Strikingly, the imaging parameter settings and scanning parameters of different CT scanners manufactured by different companies varied greatly, which may cause inconsistency in the data of radiomics model. When the image was analyzed and extracted in the digital form, the differences between extracted texture features might lead to some potential changes in the acquired images (26), which need further investigation for confirmation.

Although the AUC of the clinical indicators model was lower than that of the arterial and venous phase models, its specificity was improved as compared to the latter two models. Tumors with a large volume or a large diameter was more likely to have internal necrosis than those with a small volume. The internal necrosis of tumors exhibited uneven enhancement on enhanced CT imaging. In one study (27) investigating tumor location, size, shape, tumor growth, imaging enhancement mode and degree, tumor necrosis percentage, and distant metastasis on CT imaging in 42 patients with GISTs, it was found that the malignant degree of GIST can be predicted from the location, size, and necrosis rate of the tumor. Another study (31) evaluating 1303 patients with GISTs showed that tumor size >5 cm was significantly correlated with the increased rate of tumor recurrence. Tumor size had also been found to be of important diagnostic value in the risk classification of GISTs, irrespective of the NIH standard, AFIP standard, or AJCC staging system (32). It can be seen that the maximal diameter and internal necrosis of GISTs are significant in clinical diagnosis of potential malignancy and malignant tumors, as our study had confirmed the significant role of tumor morphology at the arterial and venous phase.

The traditional CT diagnostic criteria of radiommics showed low efficiency in the diagnosis of GISTs, with a significantly low AUC value compared with the other three models. Accurate diagnosis of the GIST tumor is closely related to the experience of the radiologists and appropriate understanding of tumor signs, especially atypical CT signs which may make differential diagnosis even more difficult.

Currently, some radiomics studies on grading the GIST malignant degree have been performed using ultrasound and magnetic resonance imaging besides CT imaging data (12, 33–39). Liu et al. (35) applied multicenter endoscopic ultrasound imaging data of 914 patients to set up a triple normalization-based deep learning framework with ultrasound-specific pretraining and meta attention (TN-USMA model) to automatically grading high- and low-risk GISTs. In comparing the diagnostic performance of one radiomics-based method and two state-of-the-art deep learning approaches, the TN-USMA model which was composed of intensity normalization, size normalization, and spatial resolution normalization achieved an overall accuracy of 0.834 (95% CI 0.772-0.885), an AUC of 0.881 (95% CI 0.825, 0.924), a sensitivity of 0.844, and a specificity of 0.832. Although the AUC of the TN-USMA model significantly outperformed the other two deep learning approaches (P < 0.05), it was less superior to our models of radiomics. Yang et al. (12) employed the magnetic resonance diffusion-weighted imaging (DWI) data of 91 patients with pathologically-confirmed GIST for radiomic model establishment and risk stratification, and the nomogram incorporating the texture signature features, maximal tumor diameter and location demonstrated a good discriminating effect of GIST malignancy with an AUC of 0.878 in the training and 0.903 in the validation group, suggesting that the texture-based model could be used to predict the mitotic index and risk potential of GISTs before surgery. Other radiomics models based on magnetic resonance imaging data of T1WI, T2WI, and ADC (apparent diffusion coefficient) had also be investigated in grading the malignant risk of GISTs (36), although with good effects in differentiating high-, intermediate- and low-risk GISTs, the AUC value was below 0.85 for T1WI, T2WI, and ADC. In radiomics models based on CT imaging data without the use of internal tumor necrosis and tumor size for evaluating the malignant risk of GISTs (33, 34, 37–39), good effects had been achieved on distinguishing high- and low-risk malignancy, but the AUC values were all below 0.90. In our study, the radiomics models using the internal tumor necrosis and tumor diameter imgaging data at the arterial and venous phases achieved an AUC value over 0.93 in both the training and validation group, suggesting a greater value of these radiomics models in differentiating the malignant risk of GISTs.

Some limitations existed in our study including the retrospective nature, Chinese patients enrolled only, a small cohort of patients at each center, and differences in the CT scanners and scanning parameters. All these issues may affect the publication bias, and the results should be explained in caution. Future studies will have to resolve these issues for better performances.

In conclusion, the morphological radiomic features of GISTs play a significant role in tumor risk stratification and can provide a reference for clinical diagnosis and treatment plan.

## Data availability statement

The original contributions presented in the study are included in the article/Supplementary Material. Further inquiries can be directed to the corresponding authors.

## Ethics statement

The studies involving human participants were reviewed and approved by Ethics committee of Affiliated Hospital of Hebei University. The patients/participants provided their written informed consent to participate in this study.

## Author contributions

JR and XY designed the study. WY, YW, LJ, and LM collected the data. WY, JR, and B-LG analyzed the data. FY supervised the study. WY wrote the original version of article. B-LG Revised the original version. All authors approved the article.

## Funding

This study was supported by the Hebei University, Health Commission of Hebei Province and Hebei Natural Fund Project(2020B05, G2019041 and 2021201017).

## Conflict of interest

Author JR was employed by General Electric Pharmaceutical (Shanghai) Co., Ltd., Shanghai, China.

The remaining authors declare that the research was conducted in the absence of any commercial or financial relationships that could be construed as a potential conflict of interest.

## Publisher’s note

All claims expressed in this article are solely those of the authors and do not necessarily represent those of their affiliated organizations, or those of the publisher, the editors and the reviewers. Any product that may be evaluated in this article, or claim that may be made by its manufacturer, is not guaranteed or endorsed by the publisher.
